# Solid Waste Management Practices and Challenges in Rural and Urban Senior High Schools in Ashanti Region, Ghana

**DOI:** 10.1155/2023/9694467

**Published:** 2023-01-31

**Authors:** Simon Boateng, Doris Boakye-Ansah, Akosua Baah, Bosco Aboagye, Prince Adu-Gyamfi Kyeremeh

**Affiliations:** ^1^Social Sciences Department, St. Monica's College of Education, P.O. Box MA, 250 Mampong-Ashanti, Ghana; ^2^Mampong Technical College of Education, P.M.B, Mampong-Ashanti, Ghana

## Abstract

This study is aimed at comparatively analyzing solid waste management practices and challenges in urban and rural senior high schools in the Ashanti region of Ghana. Multiple sampling techniques (simple random, stratified sampling, convenience sampling, stratified proportionate sampling, etc.) were used to sort 370 samples. Independent Sample *t*-test was used to compare solid waste management practices in rural and urban senior high schools. Mean and standard deviation were further used to examine the challenges the schools faced in managing waste. The study found that both rural and urban senior high schools had waste management practice systems in place but they were dissimilar. However, in both urban and rural senior high schools, the issue of inadequate resources for effective waste management was ubiquitous challenge confronting both set of schools in managing waste. Further, while poor student attitude towards waste management was a major constraint for rural schools, the urban schools had a challenge in terms of poor waste collection routine. Formation of environmental education clubs by school authorities among student can be a sine qua non for effective waste management practices among students, particularly for the rural folks. Again, waste management policies by the District Assemblies should not be exclusive to only the communities, as senior high schools have been experiencing population explosion with the introduction of the free senior high school policy.

## 1. Introduction

Sustaining effective solid waste management practices is crucial to both developed and developing countries. Waste management practices, especially the solid waste, differ significantly for developed and developing countries, for urban and rural areas, and for residential, commercial, and industrial producers [1–3]. Globally, there is a widening gap between the advanced countries and that of the developing countries regarding solid waste management [4]. For instance, in Ghana, urban domestic waste collection services are often provided by local government authorities or by private companies for a fee, while the rural residents dump their solid waste on open dumping sites for free [1].

It is noteworthy that issues of solid waste management are not only pertinent in our communities but extend from the normal resident's environment to schools as well. Even in the basic schools, the issue of solid waste cannot be overlooked, as students buy various materials that create all forms of waste [5, 6]. Water bottles, polythene bags, and other materials that bring about solid waste are found all around in the schools' environment [7, 8]. It must be noted that there has been a rapid increase in inorganic (plastic waste) waste on campuses of schools as a result of changing consumption patterns of both urban and rural dwellers [9].

For instance, in senior high schools, there is an increase in the amount of waste that is generated by students and even teachers [10]. With a population of not less than 1000 in each senior high school as a consequence of the emergence of the free senior high school policy in Ghana, there is a high level of waste generation [5, 6]. These wastes generated by students are found in the dormitories, dining halls, classrooms, and other areas on the school compound [11, 12]. These generated wastes are swept, collected, and disposed on the same environment that students are meant to have their studies [13].

Takiyudeen [14], in a research conducted on the causes of rampant cholera outbreak in various senior high schools stipulates that improper waste management system in our senior high schools is a contributing factor to the outbreak of this deadly disease. Filth is one of the causes of malaria; dumping site serves as breeding grounds for mosquitoes that are the causative agents of malaria [14, 15]. Improper waste management in various senior high schools can hinder and have negative effects on students which in turn can affect their academic life.

Notwithstanding, it is crucial to recognise that waste management practices in senior high schools may differ from one school to the other, particularly in the rural and urban dichotomy. The general waste management practices in a specific community are likely to be adopted by schools found in the community [16]. In the urban areas, people in the community collect and store waste for a waste collection organization to finally collect them at a fee [17–19]. This way of waste collection is likely to be adopted by the schools in the urban areas [18, 20, 21].

Siaw [18] asserts that the most common method of solid waste management practice in various senior high schools is dumping in pits. According to Debrah et al. [6], most of the senior high schools dig pits as storage for the waste they generate. This practice at times has various negative effects. This method brings bad smell and likely to cause breathing problems, and even at times, may create lung problems. To create a healthy and safe environment, there is the need to adopt and stick to proper waste management practices in senior high schools, since failure to manage waste well could be detrimental to students.

Meanwhile, major areas that have not received much attention when it comes to the generation of solid waste and its management are the various second cycle educational institutions in Ghana [2, 6], particularly the rural schools. Less attention is given to solid waste being generated in senior high schools. However, various senior high schools in Ghana are part of the waste generators in the country. A research conducted by Asumah [22] suggests that 3% of waste generated in Ghana is from various schools. This makes and establishes facts that waste management in various schools should be given maximum attention, especially as it has been found to link with other infectious diseases like malaria, cholera and among others [9, 23]. The urgency of the problem has caused some significant studies on waste management practices in senior high schools in urban settings [24–26]. However, the rural and urban dichotomy and dynamics largely remain novel. The study aims at comparing waste management practices in rural and urban senior high schools in the Ashanti region of Ghana.

## 2. Materials and Methods

The study adopted a quantitative approach. The quantitative research approach was used because it helped the researchers to make claims with regards to the relationships between the variable understudy. The population of the study consisted of the entire students of Armed Forces School Q and Adugyama School F in the Kumasi Metropolis and Ahafo-Ano South, respectively, in the Ashanti region of Ghana. The names of the schools have been modified for the sake of the principle of anonymity. The rationale behind restricting the population to the students of these schools was that they are in equal positions to help the researchers in getting relevant information with respect to the solid waste management practices. Again, Armed Forces School Q was chosen because of their known compliance to effective solid waste management practices ion their campus.

### 2.1. Sample and Sampling Procedures

The estimated number of students in the two schools was well above 3700, and for that reason, the sample size for this study was 370. Krejcie and Morgan's [27] formula table was used to select the 370 respondents for the study. According to Krejcie and Morgan [27], between 10% and 30% of a given population can be used for a study. Therefore, the study chose the minimum of 10% (370) sample size from 3700 students. Multiple sampling procedures (simple random, stratified, purposive, and convenience sampling techniques) were adopted in the study. The researchers used the stratified sampling technique to divide the schools into rural and urban and further divided the students into three, that is, form 1, form 2, and form 3 in their respective schools. The convenience sampling technique was used to select the school understudy. The convenient sampling technique was adopted because of the schools' proximity to the researchers, and also the Armed Forces School Q's compliance to effective solid waste management practices. The simple random sampling technique was used to select 370 students from Armed Forces School Q (250) and Adugyama School F (120). As said earlier, the schools were further put into forms 1, 2, and 3 using the stratified sampling technique for fair representation at all levels of the schools. In selecting from each stratum, the lottery method was adopted. The “Yes” and “No” responses were written on separate slip of papers and placed in a container, and the container was shaken each time a slip was picked by a student. Those who picked the “Yes” were involved. The simple random sampling technique was used for sampling because it ensured that every possible member of the population group to be sampled has an equal opportunity of being selected as part of the sample. In addition, purposive sampling technique was used to select key informants (headmaster and teachers and house masters and senior housemasters/mistresses).

To ensure that each school got a proportionate representation, proportionate sampling technique was used to select the respective sample sizes for the schools. This is represented in Table 1.

### 2.2. Data Collection Process and Tool

The researchers informed the headmasters about their intentions of carrying out a study that had to do with students and teachers on the comparative study of solid waste management practices in rural and urban schools. The respondents were assured of confidentiality and anonymity of their responses. Based on the assurances given, the student worked on their questionnaire the same day. The researcher used structured questionnaire to gather information from respondents. The questionnaire was in four sections which included, sociodemographic characteristics, which collected data on age, gender, and form of respondents; waste management practices, which collected data on the various means of disposing and collecting wastes in the various schools; health and environmental state of school, which collected data on the current health status of students in the various senior high schools; and suggestions, which collected data on key means of managing waste effectively in senior high schools.

### 2.3. Data Analysis Tools

All data collected were first edited for consistency and clarity. Afterwards, a coding format was adopted and used to effect the variable view input in the Statistical Packages for Social Sciences (SPSS) version 23 for analysis. In the meantime, all the individuals' questionnaire had been coded with the same responses having the same code numbers. The analyses conducted included descriptive statistics and regression analysis at the 0.05 level of significance. The study employed the use of an Independent Sample *t*-test to compare the waste management practices in both urban and rural schools. Finally, means and standard deviation based on four-point Likert scale responses were used to examine challenges of managing solid waste from the perspectives of the respondents.

### 2.4. Ethical Approval

The study was approved by the Committee on Human Research, Publication and Ethics of the School of Medical Sciences, Kwame Nkrumah University of Science and Technology/Komfo Anokye Teaching Hospital with reference number CHRPE/AP/317/20. Again, all participants gave verbal consent for their participation in the study.

## 3. Results

The section addresse**s** these questions based on the general objective of the study which was to comparatively analyse solid waste management practices in urban and rural senior high schools in the Ashanti region. Specifically, it looked at the sociodemographic characteristics of respondents, waste management practices, challenges to effective waste management practices, and probable solutions from the perspectives of **the** respondents from both the rural and urban senior high schools.

### 3.1. Sociodemographic Characteristics of Respondents

As part of the survey, the study collected data on the demographic characteristics of students in the selected schools. Key aspects of the demographic characteristics included age, sex, programme of study of respondents, and the form of respondents. The age of the respondents was grouped into three with a 4-year interval. This was done to enhance the identification of respondents who fell within a selected age group. Also, the programme of study was limited to four categories since these were the prevalent programmes in the schools under review. The sociodemographic characteristics of respondents considered in the survey are summarised in Table 2.

Table 2 reports that 191 (51.5%) of the respondents were males, whereas 179 (48.5%) of the respondents were females. Also, 163 (44.0%) of the respondents were less than 15 years of age, 140 (38.0%) were between the ages of 15 and 18 years, whereas 67 (18.0%) were at least 19 years old. Table 2 further reports that 74 (20.0%) of the respondents were visual arts students, 139 (37.5%) were general arts students, whereas 98 (26.5%) and 59 (16.4%) were business and general science students, respectively. The smaller number of general science students as compared to business and general arts options indicates the inherent inclination to pursue general arts and business programmes among these students. A norm which is premised on the belief that science- and mathematics-related programmes are difficult to pursue.

Finally, Table 2 indicates that 98 (26.5%) of the respondents were first year students, 113 (30.5%) were second year students, whereas 159 (43.0%) of the respondents were final years students. The higher number of second year and third years was because these were the focal group for the purposes of drawing a robust conclusion. These students had had at least a year of experience in schooling in the selected schools, so it could provide accurate data. First years were included for representativeness of the data.

### 3.2. Solid Waste Management Practices of Rural and Urban Schools

This section provides analysis towards answering, “how is solid waste managed in rural and urban senior high schools?” The researchers employed the use of an Independent Samples *t*-test to compare the waste management practices between the two schools, Armed Forces School Q (which represents the urban Population) and Adugyama School F representing the rural school. The management practices were grouped into storage, handling, and disposal. The Independent Samples *t*-test compared the mean responses of students with regards to the indicators of waste management practices based on the three indexes.  Table 3 looks at the means of storage of solid waste in the senior high schools in a five-point Likert scale as 1 = storing in plastic bag, 2 = storing in chalk box, 3 = storing in open container, 4 = storing in a dustbin, and 5 = storing in an open pile, significant at 5%.

Table 3 reports that among rural schools, wastes in the form of plastic are stored in an open pile (*M* = 4.7321, SD = 1.24473, *P* < 0.001) on the premises of the school, whilst their urban counterparts store plastic wastes in dustbins (*M* = 3.9319, SD = 1.22109, *P* < 0.001) provided at vantage points in their school. The analysis showed that at least students in senior high schools in both rural and urban areas had their respective places to store plastic waste in open containers and dustbins, respectively, before disposal.  Table 3 further reports that paper wastes are stored in dustbins provided at vantage points in the urban school (*M* = 3.7319, SD = 1.26780, *P* < 0.001), whereas the rural school stored paper wastes in open containers (*M* = 2.8521, SD = 1.17869, *P* < 0.001).  Table 3, again reports that in urban schools, food or garden wastes are kept in open containers (*M* = 3.6596, SD = 1.29226, *P* < 0.001), whereas in rural schools, food or garden wastes are stored in an open pile (*M* = 4.6423, SD = 1.6641, *P* < 0.001).

Further, Table 3 reports that cans and containers are kept in dustbins in urban schools (*M* = 3.5212, SD = 1.27892, *P* = 0.059), whereas their rural counterparts stored their can and container wastes in open containers (*M* = 2.8842, SD = 1.38351, *P* = 0.059).  Table 3 finally indicates that in terms of rags such as old and worn clothing, urban schools store them in dustbins (*M* = 3.8798, SD = 1.34055, *P* < 0.001), whereas their rural counterparts keep rags in an open pile (*M* = 4.5031, SD = 1.18560, *P* < 0.001).

### 3.3. Preference of Solid Waste Disposal Practices between Rural and Urban Schools

The study went further to make a comparison of the waste disposal methods of urban and rural schools. The comparison was based on how these students in the schools dispose off wastes with responses such as 1 = burning, 2 = indiscriminate dumping, 3 = open container, 4 = dustbin, and 5 = open pile at 5% significant level.

Table 4 reports that urban schools preferred disposing their plastic wastes in an open container (*M* = 1.4081, SD = 1.22109, *P* = 0.012) compared to rural schools who preferred burning these plastic wastes in an open pile (*M* = 2.8824, SD = 1.24473, *P* = 0.012). Table 4 again indicates that urban schools preferred disposing paper wastes in dustbins (*M* = 1.3427, SD = 1.26780, *P* < 0.001), whereas their rural counterparts preferred disposing their paper wastes through burning on open piles (*M* = 2.5142, SD = 1.17869, *P* < 0.001).  Table 3 further indicates that rural schools indiscriminately disposed off their food/garden wastes (*M* = 2.1552, SD = 1.16641, *P* < 0.001) as compared to their urban folks who preferred disposing off their food/garden-wastes in open containers (*M* = 1.4221, SD = 1.29226, *P* < 0.001).

Table 4 reports that urban schools preferred to dispose off their wastes in the form of cans and containers in open containers (*M* = 1.2312, SD = 1.27892, *P* < 0.001) compared to their rural counterparts who preferred to dispose off their cans and container wastes in open piles (*M* = 2.1381, SD = 1.38351, *P* < 0.001). Table 4 finally reports that the rural schools preferred to dispose off their rags by open burning (*M* = 2.6240, SD = 1.18560, *P* = 0.034) as compared to their urban counterparts who preferred to dispose these rags in open containers (*M* = 1.4271, SD = 1.34055, *P* = 0.034).

### 3.4. Handling of Waste in Rural and Urban Schools

The study further went on to make a comparison between the way wastes are handled in rural and urban schools using the Independent Samples *t*-test on a four-point Likert scale as 1 = male form1 students, 2 = female form one students, 3 = junior level students (both male and female), 4 = all students, and 5 = hired cleaners/labourer at 5% significant level.

Table 5 indicates that in both urban (*M* = 2.8824, SD = 1.22109, *P* < 0.001) and rural schools (*M* = 2.5821, SD = 1.24473, *P* < 0.001), junior level students are responsible for sweeping and collecting plastic waste. Table 5 reports that for paper wastes, junior students were responsible for handling them in both urban (*M* = 2.3427, SD = 1.26780, *P* < 0.001) and rural (*M* = 2.5142, SD = 1.17869, *P* = <0.001) schools. Table 5 reports again that the handling of garden/food wastes was the duty of junior level students in urban schools (*M* = 3.4221, SD = 1.29226, *P* < 0.001), whereas in the premises of their rural counterparts, the duty of handling garden/food waste was the preserve of female students (*M* = 2.1552, SD = 1.16641, *P* < 0.001). For cans and containers, urban schools employed hired hand and labourers to handle these wastes (*M* = 4.531, SD = 1.27892, *P* < 0.001), whereas rural schools left the handling of these wastes to junior level students (*M* = 2.801, SD = 1.38351, *P* < 0.001). Table 5 finally reports that hired hands and labourers were employed to handle wastes in the form of rags and worn clothing (*M* = 4.612, SD = 1.34055, *P* = 0.041), whereas in rural schools, the same duty was the preserve of junior level students (*M* = 2.624, SD = 1.18560, *P* = 0.041).

### 3.5. Challenges to Effective Waste Management Practices

This section provides an analysis towards answering the question, “what are the challenges to effective waste management in senior high schools?” The study employed the use of the Independent Samples *t*-test in this analysis. The purpose was to aid the identification of problems that are unique to rural and urban schools. A summary of the results is displayed in Table 6.

Table 6 indicates that in urban schools the attitude of students towards waste management was not a major problem affecting the effective management of waste (*M* = 1.9319, SD = 1.02139, *P* < 0.001). However, that is not the case for their rural counterparts as student attitudes were a major challenge to managing wastes effectively (*M* = 4.7321, SD =1.22031, *P* < 0.001). Table 6 reports that among urban senior high schools, the supply of waste bins was a moderate challenge (*M* = 2.5319, SD = 1.2678, *P* = 0.002), whereas the situation is a major challenge for rural senior high schools (*M* = 4.8521, SD = 1.96781, *P* = 0.002). Table 6 again indicates that in both urban (*M* = 3.6596, SD = 1.62296, *P* = 0.025) and rural (*M* = 4.6423, SD = 1.14142, *P* = 0.025) senior high schools, the issue of inadequate resources for effective waste management was ubiquitous challenge confronting both set of schools in terms of waste management. Table 6 finally reports that rural senior high schools were less affected by poor waste collection routines (*M* = 1.8842, SD = 1.38351, *P* < 0.001), whereas the impact was felt in urban senior high schools (*M* = 3.5212, SD = 1.27452, *P* < 0.001).

### 3.6. Discussions of Findings

This study examines solid waste management practices and challenges in rural and urban senior high schools in Ashanti region of Ghana. The study has established several differences that exist between rural and urban senior high schools regarding solid waste management practices and challenges that require sentient attention of policy makers. The study found that the rural senior high school stored their plastic and other forms of waste in an open pile as against their urban counterpart who stored the same wastes in either dustbins or open containers. This result may be due to the lack of clear policy planning and implementation regarding solid waste management in rural Ghana. Generally, there is an overconcentration in the urban centres regarding the effective management of solid waste. The lack of provision of dustbins in rural communities in effect has transcended to the rural schools; hence, the rural senior high schools resorting to open piles. This finding is not independent from that of Debrah et al. [6] and Gebril [2] that there are several waste management practices privy to the rural folks which include, dumping in water, mining pits, and ploughing into soil and open piles. Some of these unwholesome practices of solid waste identified during the early disposal practices still exist in senior high schools in Ghana.

Again, the rural and urban senior high schools' dichotomy regarding solid waste management was manifested in how they prefer disposing their solid waste. The study found that the urban schools preferred disposing their solid waste in an open container compared to their rural folks who preferred burning their wastes in an open pile. This finding is not quite surprising as solid waste collection services (both private and public) are abundant in the urban communities as against the rural communities, where there is almost none. In view of this, the urban senior high schools have negotiated with waste management companies like Zoomlion who have provided them with open containers and collect wastes for final disposal when they are full. Conversely, the rural senior high schools lack these services and therefore resort to disposing and burning of waste in open piles. A situation which calls for critical attention from policy makers, as it is linked to the health of students on campus. This corroborates the study carried out by Boateng et al. [1], which showed that the most common methods of solid waste disposal include dumping of waste in unregulated areas and burning of wastes on unapproved dumping sites, especially in rural areas. Liao and Li [15], in a similar way, report that waste management practice in schools is the burning of waste in open dumps.

Further, the study posits a wide difference between the handling of can waste in rural and urban senior high schools. While labourers are responsible for the handling of these wastes in urban schools, the junior students are rather responsible for the handling of the same wastes in the rural schools. Even though it is the government that employs workers for the senior high schools in Ghana, workers in all forms are skewed toward urban centres to the neglect of the rural areas, as in the case of many countries in the Sub-Saharan Africa. Again, even when the government has not given clearance for employment of labourers, the urban schools have the financial capacity to hire the services of these labourers to work for them. A situation which may give the students in urban schools some leverage in their academic pursuit, because they may have ample time for it if utilised efficiently. These findings partly contradict that of Defra [19] and Kasavan et al. [16] who posit that among urban schools the collection and handling of food waste is the preserve of hired hands and labourers.

However, the study found otherwise for the handling of plastic, paper, and food wastes to be the responsibility of the junior students (first- and second-year students). This result is maybe due to the traditional practices in senior high schools in Ghana, where first year students are responsible for cleaning the school compound. The senior students (final year students) only play supervisory role on campuses, because they hold various positions putting them in charge of such. This practice is considered to be part of the schools' training to make the students disciplined in their future endeavours.

Regarding the challenges of solid waste management practices, the study found that attitude of students in urban senior high schools towards effective waste management was not a major problem as compared to their rural folks. This may be precipitated by the fact that the school understudy was a military school, where students rigidly comply with school rules of keeping the school compound clean. Similarly, other urban schools consciously place notices at vantage point, educating and barring students and visitors from littering the compound. The situation is mostly entirely different in rural senior high schools. This finding is not different from Adeolu et al. [9] who found that in rural schools, the attitude of students is very poor and these students lack the basic instinct of appropriating wastes in appropriate cans which serves a significant challenge. Again, the study intimates that the supply of waste bins in urban schools is a moderate challenge as compared to their rural counterparts where it is a major challenge. As stated earlier, many urban schools have partnered some waste management companies like the Zoomlion which supplies them with waste bins. Even though it was occasionally, inadequate, was found not to be a major problem as in the case of the rural schools who did not have any form of partnership with a company to supply them with waste bins.

The study again indicates that the issue of inadequate resources for effective waste management is ubiquitous challenge confronting both set of urban and rural senior high schools. The introduction of the free senior high school in Ghana has increased the number of students in schools. Even though there is a glaring corresponding increase in waste generation, release of resources for effective waste management in schools may not be a matter of priority for the government. A phenomenon which is likely to ignite the spread of some infectious diseases like cholera and malaria if not attended to. This finding is profound and worrying as it corroborates [28] and Debrah et al.'s [6] studies that inadequate resources for waste management institutions to effectively collect waste affects waste management practices in schools. Finally, the study stipulates that rural senior high schools do have problems with waste collection routines compared to their urban folks. This is due to the fact that many rural schools, if not all, did not have any contract or partnership with any solid waste management company to collect waste. As a result, many of the rural schools resort to burning of these wastes in open piles, as earlier asserted by the study. On the other hand, many urban schools relied on waste management companies to collect wastes every one week. As these companies were overwhelmed with the wastes of the urban communities themselves, they were unable to collect that of the schools culminating into serious waste problems in urban schools.

### 3.7. Conclusion and Policy Implications

The purpose of the study was to comparatively analyse solid waste management practices and challenges in urban and rural senior high schools in the Ashanti region of Ghana. The study found that both rural and urban senior high schools had waste management practices system in place. However, these practices were distinctively dissimilar. While urban senior high schools had access to dustbins and containers to dispose their waste, their rural counterparts lacked these accoutrements and therefore resorted to disposing waste in open piles, a situation which had dire consequences on their health. In relation to the challenges that confronted senior high schools in effective management of solid waste, the study found that student attitudes were the major constraints for rural schools whereas for urban schools, the challenge was in terms of poor waste collection routine and adequate resources.

Formation of environmental education clubs by school authorities among student can be a sine qua non for effective waste management practices among students, particularly the rural folks. This group would help to sensitise fellow students on effective waste management practices. This peer sensitization is key, as students tend to heed to their friends when they are on campus. Waste management policies by the district assemblies should not be exclusive to only the communities as senior high schools have been experiencing population explosion with the introduction of the free senior high school. Furtherance, school authorities must encourage solid waste segregation practices among students on campus. With this, the putrescible food/garden wastes can be used for organic manure for school gardens. On the other hand, the nonputrescible wastes like plastic can be recycled for other purposes.

## 4. Limitations of the Study

Whereas longitudinal analysis migh be desirable, this study employed a cross-sectional design as opposed to a longitudinal study. This might limit the determination of any causal and temporal relationships among the various outcomes and explanatory study variables. The findings should, therefore, be taken as associations rather than being causal. It is critical to recognise that the findings of this study should be interpreted in the light of such limitations.

## Figures and Tables

**Table 1:** Sample size for each student population of sampled schools.

Schools	Student population	Relative ref.	Sample size Rf^∗^370
Armed forces school Q	2500	0.6757	250
Adugyama school F	1200	0.3243	120
Total	**3700**	**1.0000**	**370**

Source: authors' own construct, 2021.

**Table 2:** Sociodemographic characteristics of students.

Variables	Items	Frequency	Valid percentage
Sex	Male	191	51.5
	Female	179	48.5

Age	Below 15 years	163	44.0
	15–18 years	140	38.0
	19 years and above	67	18.0

Programme of study	Visual arts	74	20.0
	General arts	139	37.5
	Business	98	26.5
	General science	59	16.0

Form	First year	98	26.5
	Second year	113	30.5
	Final year	159	43.0

Source: field data (2021).

**Table 3:** Means of storage of solid waste prior to disposal.

Type of waste	Mean	Std. dev	*t*	*P* value
Plastic waste				
Urban school	3.9319	1.22109	8.151	0.001
Rural school	4.7321	1.24473		
Paper waste				
Urban school	3.7319	1.26780	6.702	0.001
Rural school	2.8521	1.17869		
Food/garden waste				
Urban school	3.6596	1.29226	6.998	0.001
Rural school	4.6423	1.16641		
Cans/container				
Urban school	3.5212	1.27892	1.893	0.059
Rural school	2.8842	1.38351		
Rags				
Urban school	3.8798	1.34055	7.123	0.001
Rural school	4.5031	1.18560		

Source: field data (2021). Means of storage: 1 = plastic bag, 2 = chalk box, 3 = open container, 4 = dustbin, and 5 = open pile. Significant at 5%.

**Table 4:** Preference of waste disposal practices between rural and urban schools.

Type of waste	Mean	Std. dev	*t*	*P* value
Plastic waste				
Urban school	1.4081	1.22109	8.151	0.012
Rural school	2.8824	1.24473		
Paper waste				
Urban school	1.3427	1.26780	6.702	0.001
Rural school	2.5142	1.17869		
Food/garden waste				
Urban school	1.4221	1.29226	6.998	0.001
Rural school	2.1552	1.16641		
Cans/container				
Urban school	1.2312	1.27892	1.893	0.001
Rural school	2.1381	1.38351		
Rags				
Urban school	1.4271	1.34055	7.123	0.034
Rural school	2.6240	1.18560		

Source: field data (2021). Means of disposal: 1 = burning, 2 = indiscriminate dumping, 3 = open container, 4 = dustbin, and 5 = open pile. Significant at 5%.

**Table 5:** Handling of waste in rural and urban schools.

Type of waste	Mean	Std. dev	*t*	*P* value
Plastic waste				
Urban school	2.882	1.22109	8.151	0.001
Rural school	2.582	1.24473		
Paper waste				
Urban school	2.343	1.26780	6.702	0.001
Rural school	2.514	1.17869		
Food/garden waste				
Urban school	3.422	1.29226	6.998	0.012
Rural school	2.155	1.16641		
Cans/container				
Urban school	4.531	1.27892	1.893	0.001
Rural school	2.801	1.38351		
Rags				
Urban school	4.612	1.34055	7.123	0.041
Rural school	2.624	1.18560		

Source: field data (2021). 1 = male form1 students, 2 = female form one students, 3 = junior level students, 4 = all students, and 5 = hired cleaners/labourer. Significant at 5%.

**Table 6:** Challenges to effective waste management.

Type of waste	Mean	Std. dev	*t*	*P* value
Student attitude				
Urban school	1.9319	1.02139	8.151	0.001
Rural school	4.7321	1.22031		
Inadequate bin supply				
Urban school	2.5319	1.26780	6.702	0.002
Rural school	4.8521	1.96781		
Inadequate resources for waste management				
Urban school	3.6596	1.62296	6.998	0.025
Rural school	4.6423	1.14142		
Poor waste collection routine				
Urban school	3.5212	1.27452	1.893	0.001
Rural school	1.8842	1.38351		

Source: field data (2021). 1 = strongly agree, 2 = agree, 3 = disagree, and 4 = strongly disagree. Significant at 5%.

## Data Availability

The raw data supporting the conclusions of this article will be made available by the authors, without undue reservation.
